# Upregulation Mitochondrial Carrier 1 (MTCH1) Is Associated with Cell Proliferation, Invasion, and Migration of Liver Hepatocellular Carcinoma

**DOI:** 10.1155/2021/9911784

**Published:** 2021-06-07

**Authors:** Guolin Chen, Shanshan Mo, Di Yuan

**Affiliations:** ^1^Department of Infectious Diseases, The First Affiliated Hospital of Harbin Medical University, Harbin, China; ^2^Pharmacy Department of Heilongjiang Sailors General Hospital, Harbin, China; ^3^Clinical Laboratory, The First Affiliated Hospital of Harbin Medical University, Harbin, China

## Abstract

Among the primary causes of cancer-associated death in the world, liver hepatocellular carcinoma (LIHC) ranks the third. LIHC is defined as the sixth most frequently diagnosed carcinoma. The gene mitochondrial carrier 1 (MTCH1) is a protein-coding gene. Recent research suggests that MTCH1 may be associated with some diseases. Here, our study attempts to explore the role and implication of MTCH1 in LIHC. Kaplan Meier Plotter and GEPIA (Gene Expression Profiling Interactive Analysis) databases were employed to determine the expression of MTCH1 and its correlation with prognostic status in LIHC patients. For the first time, our results suggested that MTCH1 was aberrantly expressed in human pan-cancer and highly expressed in LIHC. Its high expression was closely associated with metastasis of tumor, stage of cancer, and poor survival of patients. Then, through enrichment analysis, MTCH1 was found to be closely related to RNA splicing in LIHC. Subsequently, we conducted a series of functional experiments. PCR data showed that LIHC cell lines and samples are highly expressed MTCH1. CCK-8 (Cell Counting Kit-8) assays and Transwell assays indicated that silencing MTCH1 certainly suppressed cell proliferation, migration, and invasion. These findings shed the clue that MTCH1 could be regarded as the potential prognosis biomarker of LIHC and a promising therapeutic target for LIHC.

## 1. Background

As the International Agency for Research on Cancer reported, liver hepatocellular carcinoma (LIHC) is the third primary inducer amid cancer-associated death worldwide [1]. Meanwhile, LIHC is considered the sixth most diagnosed carcinoma [2, 3]. In the last few years, over 700,000 people are dying of LIHC annually, and the number is still growing every year. In the present, chemotherapy, surgical resection, and liver transplantation are effective methods for the early stage of LIHC [4]. Nevertheless, treatment strategies are limited to advanced-stage cases [5]. Compared to early primary LIHC, distant metastasis in the advanced stage is the pivotal inducer of tumor death, because LIHC is a highly aggressive and complex neoplasm disease [6–8]. No specific treatment strategy that focuses on LIHC has been developed. Thus, uncovering the hidden mechanisms in the pathogenesis of LIHC would be conducive to offering a new strategy or predictive prognostic indicator for LIHC.

The mitochondrial carrier 1 (MTCH1) is a protein-coding gene and originally described as the interactor of presenilin 1 [9]. It is also named as presenilin 1-associated protein (PSAP). MTCH1 has two widely expressed transcripts from alternative splicing. Both of them are complete mitochondrial outer membrane proteins and contain two proapoptotic domains [10]. In the absence of proapoptotic proteins, the two transcripts can induce apoptosis when overexpressed in cells [11]. Recent research suggests that MTCH1 may be associated with some diseases. For instance, Vural et al. reported that the MTCH1 expression level was associated with clinical and apoptotic parameters of neuro-Behcet's disease (NBD) [12]. Therefore, further characterization of the functional role of MTCH1 is needed.

Here, we studied the MTCH1 expression level in LIHC and its clinical implication. Also, to explore the role of MTCH1 in LIHC, we measured LIHC cell proliferation, invasion, and migration after ablating MTCH1. We first revealed the role of MTCH1 in LIHC and supplied new ideas for the treatment of LIHC.

## 2. Material and Methods

### 2.1. TNMplot Database

The database is available at http://www.tnmplot.com, including 56,938 samples from The Cancer Genome Atlas (TCGA, 394 metastatic, 9,886 tumorous, and 730 normal), gene chip-based studies (453 metastatic, 29,376 tumorous, and 3,691 normal samples), TARGET (1 metastatic, 1,180 tumorous, and 12 normal), and the Genotype-Tissue Expression (GTEx, 11,215 normal samples). In our research, we applied this database to determine the expression of MTCH1 in pan-cancer and make a comparison with MTCH1 expression profiles in normal and neoplasm tissues.

### 2.2. GEPIA Database

Gene Expression Profiling Interactive Analysis (GEPIA, http://gepia.cancer-pku.cn/index.html), functioning as an interactive web server, was applied for the analysis of RNA sequencing data from the TCGA and the GTEx projects utilizing standard processing pipeline. GEPIA offered several function analyses, containing the differential expression of neoplasm/normal samples, survival analysis of patients, profiling classified by carcinoma types or pathological stages, similar gene detection, correlation analysis, and others [13, 14]. Here, we conducted GEPIA to determine the relationship between MTCH1 expression and pathological stages and survival. Besides, we wanted to dig out MTCH1 coexpression genes.

### 2.3. The Kaplan Meier Plotter Database

The database is available at employed to evaluate 54 k gene-exerted impacts on survival in 21 types of carcinomas, comprising lung (n =3,452), breast (n =6,234), gastric (n =1,440), and ovarian (n =2,190) carcinomas [15]. The main purpose of this database is to discover and verify survival biomarkers based on a meta-analysis. The sources of the database consisted of TCGA, European Genome-phenome Archive (EGA), and Gene Expression Omnibus (GEO).

### 2.4. Enrichment Analysis

Gene Ontology (GO) enrichment analysis was used for gene annotation and biological processes (BP) analysis. Gene information in the network was analyzed by the Kyoto Encyclopedia of Genes and Genomes (KEGG) database [16–18]. For DEGs' functions and signal pathway analysis, we employed the databases for Annotation, Visualization, and Integrated Discovery (DAVID; http://david.ncifcrf.gov). *P* < 0.05 with gene counts of >5 indicated a significant statistical difference.

### 2.5. Clinical Samples

6 LIHC patients diagnosed by pathological and histological detection from our hospital were subjected to our study. All patients did not receive chemotherapy or radiotherapy before surgery. Our experiments were officially approved by the Ethics Committee of our hospital. All patients acknowledged and signed informed consents.

Additionally, the expression detail of LIHC patients was from the TCGA database (http://cancergenome.nih.gov). 419 samples were chosen in total, containing 369 LIHC samples and 50 normal samples.

### 2.6. Cell Culture

Human LIHC cell lines (Hep3B, Huh-7, BEL-7402, and MHCC-97H) and normal liver cell HL7702 were acquired from the cell bank of the Chinese Academy of Sciences (Shanghai, China) and maintained in RPMI 1640 (Gibco, USA) medium supplied by 10% fetal bovine serum (FBS, Gibco, USA) and 1% streptomycin/penicillin (Sigma-Aldrich) under 37°C humidified chamber containing 5% CO_2_ [19].

### 2.7. Cell Transfection

For transfection, siRNA of MTCH1 (si-MTCH1) was synthesized by Genepharma (Shanghai, China). Before transfection, cells were plated in 24-well plates. The next day, cells were transfected with siRNAs utilizing Lipofectamine 2000 (Invitrogen, USA) as manually instructed. Cells were reseeded and used for other studies after 48 hours of transfection. The siRNA sequences were as follows: si-MTCH1, 5′-CATCGTGCAAGTGGATGGTAAGATA-3′; si-NC, 5′-UUCUCCGAACGUGUCACGUTT-3′.

### 2.8. RNA Extraction and Quantification

The whole RNA from LIHC cells and tissues was harvested with TRIzol reagent (Invitrogen, USA) and then reversely transcribed into cDNA using RevertAid First Strand complementary DNA Synthesis Kit (Fermentas, China). qRT-PCR reaction aiming at analyzing the relative RNA expression was performed on the Rotor-Gene 3000 system (Corbett Research, Australia) with IQ SYBR Green Supermix PCR kit (Bio-Rad, USA). All experiments were carried out in triplicate. The RNA primers were as follows: MTCH1, 5′-ATCCCCTGCTCTACGTGAAG-3′ (forward), 5′-GTGAAGAAGCTCGGCAGATAG-3′ (reverse); GAPDH, 5′-CTGGGCTACACTGAGCACC-3′ (forward), 5′-AAGTGGTCGTTGAGGGCAATG-3′ (reverse).

### 2.9. Cell Proliferation

The cell proliferation ability of BEL-7402 and MHCC-97H was measured by the CCK-8 kit (Beyotime Inst. Biotech, China). Taken briefly, 1 × 10^3^ of si-MTCH1 or control-transfected cells in each well were plated in a 96-well plate. At different time incubations (0, 24, 48, 72, and 96 h), cell proliferation viability was measured by CCK8-kit. The wavelength at 450 nm was measured by a microplate reader (Bio-Rad).

### 2.10. Transwell Assay

24-well plate of Transwell chamber (Costar, USA) was taken for Transwell assay. Taken briefly, 1 × 10^5^ cells/well maintained in medium without serum were plated in the upper chambers precoated with fresh Matrigel (Corning, USA). 600 *μ*l of medium with 20% FBS was added into the lower chambers. A cotton swab was used to remove noninvaded cells. The invaded cells were washed twice by PBS and then fixed by methanol for 10 min. And then they are stained with DAPI for 10 minutes. The cells at random 5 fields were photographed under a microscope. Similar experimental procedures were performed in migration assays. The only difference was that for the migration assay, chambers needed not to precoat with Matrigel.

### 2.11. Statistical Analysis

SPSS 22.0 (Chicago, USA) and GraphPad Prism 5.0 (San Diego, USA) software were employed to analyze the data. All derived data were shown as the mean ± SD of three separate experiments in triplicate. The difference between two compared groups or among more groups was separately analyzed by Student's *t*-test and ANOVA [20, 21]. The differences existing in survival-associated curves were assessed by the log-rank test. *P* < 0.05 represented a significant statistical difference [22–24].

## 3. Results

### 3.1. Abnormal Expression of MTCH1 Was Shown in Human Pan-Cancer

There were few types of carcinomas used for the study of MTCH1 expression. Here, we employed the Kaplan Meier Plotter online tool to investigate the MTCH1 expression profile in human pan-cancer. The data revealed that MTCH1 expression was largely heightened in three types of carcinomas, containing liver carcinoma, pancreas carcinoma, and uterine carcinoma, but decreased in 13 types of carcinomas tissues, such as Acute Myeloid Leukemia (AML) and breast carcinoma (Figure 1). Our results suggested that MTCH1 expression was abnormal in human pan-cancer.

### 3.2. Diagnostic Value of MTCH1 in Liver Cancer

To analyze MTCH1 expression profiles in normal and tumor tissues, we conducted the TNMplot online tool. Gene chip and RNA-seq data displayed that, compared to normal tissues, MTCH1 expression was increased in liver carcinoma tissues (Figures 2(a) and 2(b)) (*P* < 0.001). Next, we in-depth validated MTCH1 expression in metastatic tissues, and our data indicated MTCH1 expression was greatly higher in metastatic tumor tissues, compared to that in nonmetastatic tumor tissues and normal tissues (Figure 2(c)). Tumor metastasis often means advanced tumor stage and tumor deterioration, so we analyzed the association between the expression of MTCH1 and tumor stage by the GEPIA database. As presented in Figure 2(d), the MTCH1 expression was significantly different among different cancer stages with the highest expression in stage III. Our result implied that MTCH1 was a probably useful biomarker for the diagnosis of liver carcinoma.

### 3.3. Highly Expressed MTCH1 in LIHC Exhibited an Association with Poorly Prognostic Status

To explore MTCH1 expression-exerted influence on the prognosis of LIHC patients, we conducted survival analysis for LIHC patients using the GEPIA database. It could be seen clearly from Figures 3(a) and 3(b) that, compared to LIHC patients with low expression of MTCH1, LIHC patients with high expression of MTCH1 exhibited lower overall survival (OS) rate and disease-free survival (DFS) rate. Besides, Kaplan Meier Plotter analysis showed that patients with highly expressed MTCH1 demonstrated short survival time (Figure 3(c)). These data indicated that high expression of MTCH1 presented an association with poor survival in patients with LIHC.

### 3.4. Enrichment Analysis of MTCH1 Coexpression Genes

For identifying the most likely involved biological pathways of MTCH1, we submitted coexpressed genes with MTCH1 into DAVID for GO and KEGG pathway enrichment analysis.  Figure 4(a) presents biological process terms by GO analysis. MTCH1 coexpression genes were mainly enriched in RNA splicing (via transesterification reactions), RNA splicing (via transesterification reactions with bulged adenosine as a nucleophile), mRNA splicing (via spliceosome), RNA splicing, RNA localization, and so on. In cell component terms (Figure 4(b)), those genes were mainly enriched in spliceosomal complex, catalytic step 2 spliceosome, nuclear speck, U2-type spliceosomal complex, chromosomal region, nuclear periphery, chaperone complex, nuclear envelope, ubiquitin ligase complex, and ribonucleoprotein granule.  Figure 4(c) suggests that molecular function terms primarily participated in catalytic activity (acting on RNA), single-stranded RNA/DNA binding, ubiquitin-like protein transferase activity, mRNA 3′-UTR binding, and so on. Additionally, KEGG pathway analysis (Figure 4(d)) revealed that MTCH1 coexpression genes were significantly enriched in spliceosome, RNA transport, amyotrophic lateral sclerosis, Salmonella infection, endocytosis, ubiquitin-mediated proteolysis, viral carcinogenesis, cell cycle, oocyte meiosis, and mRNA surveillance pathway. MTCH1 coexpression genes in LICH were mostly involved in the processes and pathways related to RNA.

### 3.5. Increased Expression of MTCH1 Was Shown in the Tissues and Cell Lines of LIHC

We employed TCGA database to analyze MTCH1 expression. Among 369 LIHC tumor samples and 50 normal samples, it was found that compared to normal samples, tumor samples were highly expressed MTCH1 (Figure 5(a)). To further validate that result, we additionally screened 6 pairs of LIHC samples and normal samples by PCR (quantitative reverse transcription) assays. The experimental data were the same as the findings in TCGA (Figure 5(b)). Besides, we also detected MTCH1 expression in LIHC cell lines. According to Figure 5(c), MTCH1 was upregulated in carcinoma cell lines, particularly in BEL-7402 and MHCC-97H. Our findings showed that MTCH1 probably played an important part in the progression of LIHC.

### 3.6. Knockdown of MTCH1 Suppressed the Capability of Cell Proliferation *In Vitro*

siRNAs were transfected into BEL-7402 and MHCC-97H cells to explore the impacts of reduction of MTCH1 on cell proliferation. The expression of MTCH1 mRNA was greatly reduced (Figures 5(d) and 5(e)). Subsequently, the data of CCK-8 assay detection showed that ablating MTCH1 could significantly reduce cell proliferation capability (Figures 5(f) and 5(g)).

### 3.7. Knockdown of MTCH1 Inhibited LIHC Cell Invasive and Migration Abilities

We evaluated the influence of reduced MTCH1 on cell invasion and migration by Transwell assay. Based on the results in cell lines, MHCC-97H was chosen for Transwell assays. As Figures 6(a) and 6(b) demonstrate, si-MTCH1 could significantly weaken cell migration and invasion rates. Taken together, MTCH1 might be involved in the development of LIHC and displayed as an oncogene.

## 4. Discussion

Many biomarkers have been studied in cancers [25]. Apoptosis is a way of programmed cell death [26], which is required for multicellular organism's development and internal environment stability. Apoptosis exhibits importance in the pathogenesis of several diseases [27]. However, the extent of apoptosis varies from one to another. For instance, excessive apoptosis is shown in degenerative diseases [28], while a small amount of apoptosis is in carcinoma. Actually, apoptosis is intricate and participated in various pathways. Exogenous and endogenous connections are well-studied amid apoptotic pathways [29]. The first is the response of death receptors on the plasma membrane-mediated response to external signals. The second is the transition of cells to the final executor of mitochondria. MTCH1 and MTCH2 displayed importance in the process of mitochondrial apoptosis [30]. They are named mitochondrial carrier homologs because their sequence is similar to inner membrane carriers. MTCH1 possesses two isoforms produced by alternative splicing, both of which contain two proapoptotic domains and are complete mitochondrial outer membrane proteins. Previous reports have shown that MTCH1 is vital in apoptosis, suggesting that it displays importance in carcinoma [12]. Nevertheless, it is still elusive towards the part of MTCH1 in human carcinomas. Our study for the first time explores the MTCH1 expression profile in twenty-two types of carcinomas by TNMplot databases. Bioinformatics analysis and functional verification imply that MTCH1 acts as an oncogene in LIHC.

Till now, there are few studies to validate MTCH1expression and implication in some types of carcinomas. However, in our literature, we analyzed MTCH1 expression and explored the corresponding implication in LIHC. After the analysis of MTCH1 expression in the TNMplot database and clinical samples, we found LIHC tissues and cells are highly expressed MTCH1. Additionally, our data indicated that higher expression of MTCH1 exhibited an association with metastasis of neoplasm, stage of carcinoma, and poor survival of LIHC patients. Our data implied that MTCH1 expression was a probable indicator of LIHC patients' prognosis. Subsequently, we carried out GO and KEGG enrichment analysis to explore the function and the mechanism of MTCH1 involved in LIHC. The results suggested that MTCH1 possibly participates in the regulated process of RNA splicing in LIHC.

As we all know, RNA splicing is an extensive process that causes a transcriptional variation of structural and the diversity of proteomic [31]. Deregulated splicing occurs in carcinomas, resulting in various products with function and nonfunction. The events from cancer-specific splicing easily promote the development of disease [32]. Abnormal splicing exerts an effect on many carcinomas and brought about multiple features. Apoptosis and metastasis could be influenced by alternative splicing of numerous genes [33]. For instance, BCL2L1 (BCLXL), as a transcript variant of anti-apoptotic protein, is highly expressed in carcinoma and resistant to apoptosis [34]. Transcripts from abnormal TP53 splicing showed a relationship with apoptosis and proliferation. The above-mentioned studies suggest that abnormal splicing widely occurred in carcinomas, and MTCH1 might affect LIHC progression via RNA splicing.

Finally, we assessed the impacts of reduced MTCH1 on LIHC cell metabolism. The results demonstrated that reducing MTCH1 powerfully suppressed MHCC-97H and BEL-7402 cell proliferation, invasion, and migration. Our data collectively revealed that MTCH1 was displayed as an oncogene and functioned crucially in the oncogenesis and development of LIHC.

This study has some limitations. First, the number of clinical samples is not large enough. In future research, we will collect more LIHC clinical samples to detect MTCH1 gene expression and MTCH1 protein expression. Second, we plan to analyze the function of MTCH1 in animal models in subsequent studies.

## 5. Conclusions

Based on multiple public databases, we analyzed the high expression of MTCH1 in LIHC, and its high expression is closely related to tumor metastasis, tumor staging, and poor patient quality of life. Highly expressed MTCH1 was found in LIHC samples and cell lines. The unsatisfying prognosis of LIHC patients was also found to be related to high MTCH1 expression. Besides, our findings suggested that MTCH1 facilitated LIHC cell proliferation, invasion, and migration. We have revealed for the first time that MTCH1 may play a role in the occurrence and development of LIHC. Collectively, our findings suggested that MTCH1 was a promising prognosis factor and therapeutic target for LIHC, providing new and useful information for the study of the mechanism of LIHC.

## Figures and Tables

**Figure 1:** To analyze MTCH1 mRNA level in human pan-cancer by online tool TNMplot. N indicates normal tissues, and T represents tumor tissues. Significant differences by the Mann–Whitney *U* test between normal and tumor tissues were marked with red. ^∗^*P* < 0.05.

**Figure 2:** Diagnostic value of MTCH1 in liver cancer. (a) Violin plots of the expression of MTCH1 in liver normal and tumor tissues based on gene chip data of TNMplot. (b) Violin plots of the expression of MTCH1 in liver normal and tumor tissues based on RNA microarray data of TNMplot. (c) Violin plots of the expression of MTCH1 in liver normal, tumor, and metastatic tissues based on gene chip data of TNMplot. (d) Box plots of MTCH1 gene expression in different liver cancer stages based on the GEPIA database.

**Figure 3:** Analysis of the association between the prognostic value and MTCH1 expression in liver carcinoma. (a) GEPIA database analysis of OS curve of LIHC patients with highly expressed or lowly expressed MTCH1. (b) GEPIA database analysis of DFS curves of LIHC patients with highly expressed or lowly expressed MTCH1. (c) Kaplan Meier Plotter database analysis of OS curves of LIHC patients with highly expressed or lowly expressed MTCH1.

**Figure 4:** Enrichment analysis of MTCH1 coexpression genes, with the GO biological process (a), cell component (b), molecular function (c), and KEGG pathway (d). GO: Gene Ontology; BP: biological process; CC: cellular component; MF: molecular function; KEGG: Kyoto Encyclopedia of Genes and Genomes.

**Figure 5:** MTCH1 expression was raised in the tissues and cell lines of LIHC. (a) Analysis of MTCH1 expressions in LIHC tumor and normal samples in TCGA database. (b) To analyze MTCH1 expressions in 6 pairs LIHC tumor and normal liver samples. (c) Assessment of MTCH1 expressions in LIHC cell lines and normal liver cell lines. (d, e) Detection of MTCH1 mRNA expression in BEL-7402 and MHCC-97H cell lines transfected with si-MTCH1. (f, g) Si-MTCH1 suppressed cell proliferation in BEL-7402 and MHCC-97H. ^∗^*P* < 0.05.

**Figure 6:** Knockdown of MTCH1 inhibited the invasive and migration abilities of LIHC cells. (a, b) Analysis of cell migration and invasion ability in siRNA-transfected MHCC-97H. ^∗^*P* < 0.05.

## Data Availability

The expression detail of LIHC patients was from the TCGA database (http://cancergenome.nih.gov).
